The article "Effects of Plyometric Exercises versus Flatfoot Corrective Exercises on Postural Control and Foot Posture in Obese Children with a Flexible Flatfoot" was retracted in 2023. Reasons: signs of a paper mill; suspected computer-generated content; unreliable results or conclusions; concerns about the data.

# Effects of Plyometric Exercises versus Flatfoot Corrective Exercises on Postural Control and Foot Posture in Obese Children with a Flexible Flatfoot

**DOI:** 10.1155/2021/3635660

**Published:** 2021-10-31

**Authors:** Hatem H. Allam, Alsufiany Muhsen, Mosfer A. Al-walah, Abdulmajeed N. Alotaibi, Shayek S. Alotaibi, Lamiaa K. Elsayyad

**Affiliations:** ^1^Department of Physical Therapy, College of Applied Medical Sciences, Taif University, Saudi Arabia; ^2^Faculty of Physical Therapy, Misr University for Sciences and Technology, Egypt; ^3^Children Hospital, Taif Health Affairs, Ministry of Health, Saudi Arabia; ^4^Department of Medical Rehabilitation and Physiotherapy, Children Hospital, Ministry of Health, Taif, Saudi Arabia; ^5^Department of Biomechanics, Faculty of Physical Therapy, Cairo University, Egypt

## Abstract

**Background:**

Obesity contributes to the acquired flatfoot deformity which in turn impairs balance.

**Aim:**

The purpose of the current study was to compare the effect of plyometric exercises with flatfoot corrective exercises on balance, foot posture, and functional mobility in obese children with a flexible flatfoot.

**Methods:**

Forty-seven children participated in the study. Their age ranged from 7 to 11 years. Participants were randomly divided into 3 groups: experimental group I (EGI), experimental group II (EGII), and the control group (CG). The EGI received plyometric exercises and the EGII received corrective exercises, 2 sessions weekly for 10 weeks. The control group did not perform any planned physical activities. The Prokin system was used to assess balance, the timed up and go test (TUG) was used to assess functional mobility, and the navicular drop test (NDT) was used to assess foot posture.

**Results:**

EGI showed significant improvement in all balance parameters, foot posture, and TUG. EGII showed improvement in the ellipse area and perimeter in addition to foot posture and TUG.

**Conclusion:**

Plyometric exercises and foot correction exercises had a positive effect on foot posture, balance, and functional mobility in obese children with flatfeet.

## 1. Introduction

Obesity appeared among children and adults as one of the critical and major community health worries within the past century [1]. The prevalence of childhood obesity has been noticed over the last 3 decades [2]. Moreover, obesity also affects all daily living activities like walking or standing skills and negatively affects balance and ability to alter positions. Additionally, it is one of the main factors that causes an acquired flat foot deformity which in turn impairs the balance strategy [3]. Balance is considered as multiple processes that require mechanical, sensory, and kinetic elements of motion to be coordinated. It may be negatively influenced by many factors such as sensory impairment, abnormal muscle response, poor muscle strength, and the presence of certain foot abnormalities such as a flatfoot [4]. Some studies have confirmed that the impaired balance may affect the quality of life, many skills, and many daily living activities in children and adults [5].

Riccio et al., [6] mentioned that rehabilitation therapy, which includes the constant proprioceptive stimulation of the foot, is likely to achieve improvement in the plantar arch and correct the flexible flatfoot. Additionally, there is evidence that exercises have a crucial role in improving balance. It strengthens the muscles that enhance balance, walking ability, and correct deformities [7]. Published research has demonstrated that balance has improved by applying certain stretching procedures, proprioceptive stimulation techniques, and strengthening exercises [8]. One of the approaches that enhance balance in children is plyometric exercises [9]. Plyometric exercise indicates a quick and strong interaction movement between both eccentric and concentric contractions [10]. This type of exercise is secure and efficient in adults and children for enhancing balance, jumping skills, reaction time, bone mineral density, endurance, muscle power and strength, energy production, motor performance, and coordination [11]. Certain studies concluded that there were some improvements in postural stability after the application of a 15-minute plyometric exercise [12]. To date, little is known about the effect of plyometric exercises on foot posture in obese children with flexible flatfeet. Thus, the purpose of the current study was to compare the effect of plyometric exercises with flatfoot-corrective exercises on balance, foot posture, and functional mobility in obese children with a flexible flatfeet. The current study could help the obese children to benefit from the different exercise protocols which may contribute to improvements in their quality of life.

## 2. Materials and Methods

### 2.1. Study Setting

The study was conducted at the balance lab of the Faculty of Applied Medical Sciences. It was started on 15 January 2021.

### 2.2. Subjects

A sample of 47 male children participated in the current study without having female participants due to the cultural issues and order of the society in Saudi Arabia. The sample size was detected by using statistical power analysis—*G*∗power (power, 0.85; *α* = 0.05; effect size = 0.5, Pillai *V* = 0.2). The participants were selected randomly from different elementary schools in Taif, Saudi Arabia. Participants were enrolled by contacting their parents by phone using the phone numbers in the schools' database. Their age ranged from 7 to 11 years. Initially, a specialist examiner conducted a comprehensive evaluation of all participants. He was blinded about the groups' division. Inclusion criteria are as follows: all children were classified as obese (their body mass index percentile is equal to or greater than the 95th percentile). The participants were not involved in strength, balance training, or competitive sports aiming to enhance muscular strength or balance. All participants had balance impairments and a mobile flat foot. Their degree of flatfoot deformity according to NDT was ranged from 16 to 19 millimeters in all participants. The exclusion criteria were as follows: the children were excluded when they had a previous injury to the lower limb which required medical care or had other confounding conditions, such as deformity of or surgery in the lower limb or visual impairment. Additionally, they were excluded if they engaged in obesity treatment programs three months prior to the study. The written informed consent (from parents or children's guardians) was obtained before they enrolled in the study.

### 2.3. Randomization

A simple randomization technique was used. After gathering the baseline measurements, the participants were randomly assigned into three groups: experimental group I (EGI) contained 16 participants, experimental group II (EGII) contained 16 participants, and the control group (CG) contained 15. The stratification was done using sealed envelopes. The children were not aware of the group that they belonged to.

Demographic data collection was as follows: a specially designed survey was used to collect demographic data for all participants such as age, weight, and height.

### 2.4. Body Mass Index Percentile for Boys

BMI percentile is a screening tool used to classify the participant's degree of obesity in children according to the American Academy of Pediatrics recommendations. To calculate the BMI percentile, at first, obtain accurate height and weight measurements for each child. The subjects' body weight in bare feet and with minimal clothing was measured. Standing height was measured with the children standing straight without footwear. The height and weight were measured twice to minimize errors. The body mass index (BMI)was then calculated by dividing the weight (kg) by height (m) squared.

### 2.5. Balance Assessment

The static balance was assessed by using the Prokin system (PK 252, TecnoBody S.r.l., Italy). The balance assessment is based on the degree of postural sway using a tilting board. Before the actual assessment, all participants were engaged in certain practical sessions and the whole procedures were illustrated to them to be familiarized with the testing procedures and balance device.

#### 2.5.1. Starting the Test

In the first step, the system was opened and calibrated and the demographic data was entered (name, age, height, and weight). The next step is selecting the type of stability test, and the participant stands comfortably on the tilting board and was asked to look towards at the screen keeping his hands beside the body while his eyes are focused on the fixed target on the screen. Each participant applied three trials with eyes opened (EO) and the mean score was recorded. The participants had a five-minute break after each trial, and we tried to avoid any distractions. There are four variables that were measured for all participants at the beginning and at the end of the study with EO: perimeter area (mm), ellipse area (mm^2^), standard backward-forward deviation, and standard medial-lateral deviation.

### 2.6. The Navicular Drop Test

(NDT) was used to assess the degree of flatfoot deformity. The NDT revealed excellent reliability, with ICC values reaching 0.945 and standard error of measurement < 1 mm [13]. Firstly, the subtalar neutral position was accustomed while the child was in the sitting position with both hips and knees at 90°, and then, the navicular tuberosity was palpated and marked. The distance between the navicular tuberosity and the floor was measured in millimeters using a stainless-steel high-accuracy electronic digital display slide caliper. After that, the participant was instructed to stand in a relaxed foot posture and the navicular tuberosity was palpated and marked again to avoid any error due to skin shifting and then the height of the mark measured from the floor. The ND was the difference in the navicular tuberosity height between both marks [14].

### 2.7. Functional Mobility

Functional mobility was assessed using the timed up and go (TUG) test to detect participants' functional mobility. It is a valid and reliable test. At first, a sign was placed 3 meters away from the chair. A seat with back support without arms was chosen from the children's environment. The seat should allow the feet to be flat on the ground and the knee and hip to bend 90 degrees. Then, the child was asked to stand up, walk at his free gait, touch the mark, and return to sit down on the chair. The time was counted as the child left the seat and stopped when the child returned to the sitting position using a stopwatch. The test was run three times and the average value was taken [15].

### 2.8. The Intervention

The EGI received a plyometric exercise program. The EGII received the corrective exercises. The control group was not involved in any planned physical activity during the intervention period but persisted in their traditional physical activities. The designed exercises were applied two sessions per week with three days of rest in between for 10 weeks. The session started with 5 minutes warming up and ended with 5 minutes cooling down in the form of gentle stretching of the lower limb muscles. All participants were engaged in certain practical sessions at the beginning of the study to be familiarized for all intervention procedures. Additionally, the supervisor emphasized the correct application of the exercises. The selected plyometric exercises and their repetitions are illustrated in Table 1 according to Johnson et al. [16]. It was done on a spongy mat for shock absorption. We emphasized that all participants should get down from jumping on tiptoes and the weight-bearing activities should be done with foot pronation control. The jumps were divided into five sets and two-minute rests were given in between each set and the other. The selected corrective exercises and activities are illustrated in Table 2 according to Riccio et al. [6].

### 2.9. Ethical Considerations

The ethical committee at the research and studies department, directorate of health affairs, Taif, Saudi Arabia (IBR registration number with KACST, KSA HAP-02-T-067), approved the current study on 11 November 2020 with approval number 452.

### 2.10. Study Design and Data Analysis

A randomized controlled trial was used to investigate the effect of plyometric exercises with flatfoot-corrective exercises on balance, foot posture, and functional mobility in obese children with flexible flatfoot. This was a randomized clinical trial of the parallel-group design. The study was registered and posted on the Clinical Trials.gov public website with ID (NCT05026294). The study was double blinded, the examiners and participants were blinded about the group division. All statistical measures were performed through the Statistical Package for Social Studies (SPSS) version 26 for Windows. The MANOVA test was conducted to determine if there were any significant differences in the mean values of age, weight, height, and BMI between both groups. Additionally, repeated measures MANOVA was used to compare the within- and between-subject effects of both interventions (Table 3). The alpha level was set at 0.05.

## 3. Results

### 3.1. Baseline Comparison

There were no significant differences among the three groups at the beginning of the study either in the demographic data or in the study variables (Table 4).

### 3.2. Postintervention (within-Subject Comparisons)

The EGI showed a significant improvement in all assessed balance parameters (ellipse area, perimeter, backward-forward deviation, and mediolateral deviation) in addition to the significant improvement in foot posture (as indicated by navicular height) and TUG. Regarding EGII, there was a significant improvement in the previous items except for the backward-forward deviation and the mediolateral deviation which showed nonsignificant improvement. On the other hand, there were no significant changes in the CG (Table 5).

### 3.3. Postintervention (between-Subject Comparison)

Concerning EGI, it showed a significant difference in all assessed parameters when it was compared to the EGII and CG except the improvement in foot posture and TUG which showed a nonsignificant difference between EGI and EGII. EGII showed significant improvement in all parameters when compared to the CG except for the backward-forward deviation which showed nonsignificant improvement in the EGII (Table 6).

## 4. Discussion

The study is aimed at investigating the effect of plyometric exercises on foot posture, balance, and functional mobility in obese children with mobile flatfeet. We have selected the balance parameters to be investigated in obese children because appropriate balance control is necessary for routine activities of daily living and obesity has a tremendous negative effect on balance [17]. The results of the study revealed that there was significant improvement in all balance parameters, foot posture, and TUG in EGI. EGII showed improvement in the ellipse area and perimeter in addition to foot posture and TUG without improvement in the backward-forward and mediolateral deviation.

Concerning preintervention balance assessment, the results of the study revealed that obese children have deficient balance skills. This comes in agreement with Deforche et al. [18] who mentioned that obese prepubertal males have decreased both static and dynamic balance and postural skills. Moreover, obese children have deficits in the torque of the ankle muscles needed for stability when they are subjected to any oscillations [17]. Additionally, deficits in balance strategies in obese children preintervention had impaired functional mobility as represented by the TUG test score [18].

Concerning the effect of plyometric exercises on balance, the results of the current study revealed that the balance was improved significantly in the EGI postintervention. This comes in consistency with Arazi and Asadi [19] who mentioned that muscle strength and balance skills were improved after 8 weeks of aquatic and land plyometric exercises in young athletes. Moreover, Myer et al. [20] mentioned that the balance performance was improved after the application of the plyometric training program. Additionally, Chaouachi et al. [21] were in line with our findings when they reported that plyometric training improved balance, jumping skills, and squat strength measures like the combined training program. The improvement in balance skills after plyometric exercises may be related to the rapid stretch-shortening cycle and combines shifts of the center of gravity in both vertical and horizontal directions that may improve postural control and equilibrium [22]. Furthermore, enhanced cocontraction of the lower extremity muscles and the improvement in proprioception and neuromuscular control after plyometric training played a role in balance improvement [23].

On the other hand, Twist et al. [24] contradict our findings when they mentioned that unilateral balance performance was impaired 24 hours after plyometric exercise. This contradiction may be related to fact that they had used a high-intensity plyometric exercise program (200 jumps per session). They reported that this designed intensive plyometric program may induce symptoms of muscle damage and muscle soreness that negatively affected the balance performance.

Concerning the effect of plyometric exercises on foot posture, the results of the current study revealed that there was a significant improvement in the foot posture in EGI after plyometric training. We can attribute this improvement to the improvement in plantar flexor strength and mechanical properties after plyometric exercises. Kubo et al. [25] support this idea when they found a significant increase in plantar flexor muscle activity during the concentric phase of vertical jumps. Furthermore, the results obtained by Kyröläinen et al. [26] denoted a significant improvement in both maximum voluntary contraction and muscular activity and strength of plantar flexors after plyometric exercises. Moreover, Weist et al. [27] confirmed the relation between the plantar flexors and the medial longitudinal arch (MLA) when they concluded that fatigue of plantar flexors reduces its supination action and increases foot pronation. Additionally, Fourchet et al. [28] found that decreased calf muscle activity due to fatigue was associated with an increase in the contact area under the MLA. Kamalakannan and Swetha [29] came in agreement with our results when they concluded that robe skipping activities improved the foot arch and functional activities of the lower limb.

On the other hand, Klaikaew and Panichaporn [30] contradict our results when they reported dropping down of the navicular and a decrease in the height of the MLA after repetitive hopping. However, they used a vigorous hop technique (hopped 60 times/minute/set for 3 sets with 30 sec walking after each set). They related the navicular drop to muscle fatigue after exercise.

Concerning the effect of corrective exercises on the foot arch, the results of the study revealed that there was a significant improvement in the foot posture in EGII postintervention. Halabchi et al. [31] confirmed our findings when they have stated that the use of a suitable rehabilitation program may improve the flexible flatfoot posture in children. Their rehabilitation program included flexibility, strength, and proprioceptive training exercises which come in consistency with our corrective exercise program. Furthermore, Riccio et al. [6] agreed with our results when they mentioned that rehabilitation therapy, which depends on the constant proprioceptive stimulation of the foot, is likely to achieve improvement in the plantar arch and correct the calcaneovalgus deformity in a flexible flatfoot. The proprioceptive training is essential in the improvement of the reflex circuits, which is vital for proper confidence in both static and dynamic foot placements, which in turn improves balance and functional mobility. On the other hand, Namsawang et al. [32] contradict our results as they found that exercises for foot muscles did not improve the ND. Their results may be due to the short duration of the program (only 4 weeks) that is considered as one of their study's limitations.

Concerning the effect of corrective exercises on balance, the results of the study revealed that there was a significant improvement in all balance measures in EGII postintervention except for the backward-forward and mediolateral deviation. The improvement in the balance measures may be attributed to an increase in the strength of the intrinsic muscles of the foot, which in turn improves the arch height and postural control as reported by Kim and Kim [33]. Moreover, Sudhakar et al. [34] added that the runners with low arches had less balance than those with normal arches, which means that the increase in the arch height improves the balance strategy.

Regarding the improvement in functional mobility, the results of the current study showed that there was a significant improvement in the TUG test scores in both EGI and EGII when it was compared with CG at the endpoint. The improvement may be related to the improvement in balance skills, muscle strength, and foot posture that occurred in both experimental groups.

### 4.1. Limitations

Only male children were examined without having female participants because of cultural values in Saudi Arabia. Additionally, foot posture was assessed using the ND test only.

## 5. Conclusion

Both plyometric exercises and foot correction exercises had a positive effect on foot posture, balance, and functional mobility in obese children with flatfeet. Both should be considered in the rehabilitation of children with obesity.

## Figures and Tables

**Table 1:** The repetition of plyometric exercises during the intervention period.

The exercise	Repetitions				
	Weeks 1 and 2	Weeks 3 and 4	Weeks 5 and 6	Weeks 7 and 8	Weeks 9 and 10
Jump jacks	6	7	8	9	10
Skipping	8	9	10	11	12
Jump side to side	6	7	8	11	12
Jump front and back	6	8	10	11	13
Vertical jump	6	8	10	11	13
Hopping forwards and backwards on the right foot	6	7	8	9	10
Hopping forwards and backwards on the left foot	6	7	8	9	10
Short jump forwards and backwards	6	7	8	9	10
Total repetitions	50	60	70	80	90

**Table 2:** Corrective exercises and activities for the flexible flatfoot adopted from Riccio et al. [6].

Aim	Exercises and activities
Flexibility	Passive range of motion exercises and global movement of the ankle and all foot joints; stretching of the calf and peroneus brevis muscles
Strengthening, proprioception, and balance	Anterior and posterior tibialis muscles and the flexor hallucis longus (to neutralize valgus), intrinsic, interosseus plantaris muscles, and the abductor hallucis (to prevent anterior arch flattening); global activation/movement of the muscles involved in maintaining the medial longitudinal arch and the varus; single-leg weight bearing (with pronation control); toe and heel walking; descending an inclined surface

**Table 3:** MANOVA results for the study variables.

Effect	Test	*F*	*P*
Variables∗groups	Wilks' lambda	3.384	0.000
Time∗groups		7.477	0.000
Variables∗time		13.952	0.000
Variables∗time∗groups		6.693	0.002

**Table 4:** Bonferroni pairwise comparisons for demographic characteristics and the study variables of the three groups at the beginning of the study.

Variables	*M* ± SD			MD					
	EGI	EGII	CG	EGI-EGII	*P*	EGI-CG	*P*	EGII-CG	*P*
Age	9.48 ± 1.12	9.74 ± .95	9.07 ± 1.22	−0.27	1	0.407	0.92	0.67	0.28
Weight	45.37 ± 8.14	41.44 ± 6.02	42.04 ± 8.55	3.93	0.46	3.34	0.69	−0.60	1
Height	1.37 ± .17	1.35 ± .14	1.25 ± .12	0.022	1	0.12	0.09	0.09	0.24
BMI	23.71 ± 2.06	22.71 ± 3.06	22.01 ± 2.05	1.003	0.76	1.7	0.18	0.69	1
Ellipse area	529.64 ± 81.35	614.05 ± 125.58	581.02 ± 184.98	−84.41	0.26	−51.38	0.89	33.03	1
Perimeter	706.33 ± 170.5	631.33 ± 192.22	570.13 ± 112.99	75.001	0.6	136.2	0.074	61.2	0.9
BFD	7.96 ± 1.5	8.62 ± 1.4	7.95 ± 1.93	−0.67	0.76	0.001	1	0.67	0.78
MLD	4.64 ± 1.16	4.03 ± 1.03	4.07 ± 1.39	0.61	0.48	0.56	0.59	−0.043	1
ND	17.25 ± 3.55	16.94 ± 1.81	18.47 ± 2.9	0.31	1	−1.21	0.72	−1.53	0.43
TUG	7.53 ± .58163	7.26 ± .397	7.27 ± .36	0.27	0.31	0.26	0.37	−0.011	1

EGI: experimental group 1; SD: standard deviation; MLD: mediolateral deviation; EGII: experimental group 2; MD: mean difference; ND: navicular drop test; CG: control group; *M*: mean; TUG: time up and go test; BFD: backward-forward deviation.

**Table 5:** Bonferroni pairwise comparisons for within-subject effect.

Variables	EGI				EGII				CG			
	*M* ± SD		MD	*P*	*M* ± SD		MD	*P*	*M* ± SD		MD	*P*
	Pre	Post			Pre	Post			Pre	Post		
EA	529.64 ± 81.35	401.02 ± 98.98	128.62	0.012	614.05 ± 125.58	504.99 ± 105.44	109.05	0.031	581.02 ± 184.98	616.47 ± 99.4	−35.45	0.487
PR	706.33 ± 170.5	449 ± 75.08	257.32	0.000	631.33 ± 192.22	531.17 ± 102.45	100.16	0.022	570.13 ± 112.99	619.71 ± 84.99	−49.58	0.260
BFD	7.96 ± 1.5	6.6 ± 1.43	1.34	0.024	8.62 ± 1.4	8.2 ± 1.27	0.42	0.463	7.95 ± 1.93	8.47 ± 1.35	−0.52	0.386
MLD	4.64 ± 1.16	2.9 ± 0.54	1.74	0.000	4.03 ± 1.03	3.35 ± 0.56	0.68	0.054	4.07 ± 1.39	4.21 ± 0.39	−0.14	0.698
ND	17.25 ± 3.55	13.69 ± 1.49	3.56	0.000	16.94 ± 1.81	14.63 ± 1.96	2.31	0.006	18.47 ± 2.9	17.73 ± 1.16	0.73	0.381
TUG	7.53 ± 0.58	8.44 ± 0.64	−0.91	0.000	7.26 ± 0.4	8.68 ± 0.72	−1.41	0.000	7.27 ± 0.36	7.15 ± 0.43	0.13	0.344

EGI: experimental group 1; SD: standard deviation; PR: perimeter; EGII: experimental group 2; MD: mean difference; BFD: backward-forward deviation; CG: control group; EA: ellipse area; MLD: mediolateral deviation; *M*: mean; ND: navicular drop test; TUG: time up and go test.

**Table 6:** Bonferroni pairwise comparisons for between-subject effect.

Variables	*M* ± SD			MD					
	EGI	EGII	CG	EGI-EGII	*P*	EGI-CG	*P*	EGII-CG	*P*
Ellipse area	401.02 ± 98.98	504.99 ± 105.44	616.47 ± 99.4	−103.97	0.017	−215.44	0.000	−111.47	0.011
Perimeter	449 ± 75.08	531.17 ± 102.45	619.71 ± 84.99	−82.17	0.035	−170.7	0.000	−88.53	0.023
BFD	6.62 ± 1.43	8.2 ± 1.27	8.47 ± 1.35	−1.579	0.006	−1.85	0.001	−0.28	1.0
MLD	2.9 ± 0.54	3.35 ± 0.56	4.21 ± 0.39	−0.449556	0.047	−1.31	0.000	−0.86	0.000
ND	13.69 ± 1.49	14.63 ± 1.96	17.73 ± 1.16	−0.938	0.302	−4.05	0.000	−3.11	0.000
TUG	8.44 ± 0.64	8.68 ± 0.72	7.15 ± 0.43	−0.237	0.840	1.29	0.000	1.53	0.000

EGI: experimental group 1; SD: standard deviation; MLD: mediolateral deviation; EGII: experimental group 2; MD: mean difference; ND: navicular drop test; *M*: mean; BFD: backward-forward deviation; TUG: time up and go test.

## Data Availability

The data used to support the findings of this study are available from the corresponding author upon request.

## Supplementary Materials

Supplementary Materials The CONSORT 2010 checklist was provided.
